RETRACTED

# Andrographolide Alleviates Oxidative Damage and Inhibits Apoptosis Induced by IHNV Infection via CTSK/BCL2/Cytc Axis

**DOI:** 10.3390/ijms25010308

**Published:** 2023-12-25

**Authors:** Qi Liu, Linfang Li, Jingzhuang Zhao, Guangming Ren, Tongyan Lu, Yizhi Shao, Liming Xu

**Affiliations:** 1 Heilongjiang River Fisheries Research Institute, Chinese Academy of Fishery Sciences, Harbin 150070, Chinazhaojingzhuang@hrfri.ac.cn (J.Z.); renguangming@hrfri.ac.cn (G.R.); lutongyan@hrfri.ac.cn (T.L.);; 2 Key Laboratory of Aquatic Animal Diseases and Immune Technology of Heilongjiang Province, Harbin 150070, China

**Keywords:** IHNV, andrographolide, oxidative stress, apoptosis, antiviral drug

## Abstract

Infectious hematopoietic necrosis virus (IHNV) is an important pathogen that causes significant economic losses to salmon trout farming. Although vaccines have been invented for the treatment of IHNV, findings from our previous survey show that breeding enterprises and farmers require effective oral drugs or immune enhancers. However, studies on the development of oral drugs are limited. In the present study, we used bioinformatics methods to predict the protein targets of andrographolide (Andro) in IHNV. Cells were infected with IHNV, and the effect of andrographolide was explored by evaluating the expression levels of genes implicated in oxidative stress, activities of antioxidant enzymes, and the expression of genes implicated in apoptosis and necrosis. In the present study, cells were divided into NC, IHNV, IHNV+10 μM andrographolide, and IHNV+20 μM andrographolide groups. qRT-PCR was performed to determine the expression level of genes, and an antioxidant enzyme detection kit was used to evaluate the activities of antioxidant enzymes. Fluorescent staining was performed using a reactive oxygen species detection kit (ROS) and Hoechst 33342/PI double staining kit, and the mechanism of alleviation of apoptosis and oxidative stress andrographolide after IHNV infection was determined. The results indicated that andrographolide inhibits viral growth by binding to the NV protein of IHNV and increasing the antioxidant capacity of the body through the CTSK/BCL2/Cytc axis, thereby inhibiting the occurrence of IHNV-induced apoptosis. This is the first study to explore the antagonistic mechanism of action of andrographolide in alleviating IHNV infection. The results provide valuable information on alternative strategies for the treatment of IHNV infection during salmon family and provide a reference for the use of andrographolide as an antioxidant agent in agricultural settings.

## 1. Introduction

Andrograpis paniculata is a traditional Chinese medicinal plant that is used for the treatment of various diseases. Andrographolide is a diterpenoid lactone compound isolated from Andrograpis paniculate and is the main active ingredient of graprographia [1,2]. Andrographolide’s molecular formula is C_20_H_30_O_5_; the chemical name is 2(3H)-Furanone, 3-[2-[(1 r, as 4, 5 r, 6 r, 8 as)-decahydro-6-hydroxy-5-(hydroxymethyl)-5, 8-dimethyl-2-a methylene-1-naphthalenyl]ethylidene]dihydro-4-hydroxy-, (3E,4S). The chemical structure diagram is in Figure S1. The compound is soluble in boiling ethanol, slightly soluble in methanol or ethanol, slightly soluble in chloroform, and insoluble in water. In recent years, many Asian and European researchers have begun to study the activity, safety, and efficacy of andrographolide, confirming its practical value in production and daily life. Andrographolide has anti-inflammatory and antibacterial activities, which have protective effects on the liver, heart, and nervous system. Moreover, the compound plays an important role in various diseases such as jaundice, bronchitis, cardiovascular diseases, and skin diseases [3,4,5]. In addition, the progression of non-small cell lung cancer [6], breast cancer, gastric cancer, and colon cancer [7] can be inhibited by andrographolide through the promotion of autophagy, alleviation of anti-tumor immunosuppression, and macrophage polarization.

RETRACTED

Infectious hematopoietic necrosis (IHN) is an acute infectious disease that affects fishes and is caused by the infectious hematopoietic necrosis virus (IHNV), which is highly common in salmonids. IHN can cause 90 to 100% mortality in rainbow trout (*Oncorhynchus mykiss*) depending on differences in host species, virus strains, and environmental conditions [8,9]. Based on the significant economic losses caused by infectious hematopoietic necrosis to the global rainbow trout aquaculture industry each year, the World Organization for Animal Health (OIE) listed it as an animal disease that must be declared during import and export. IHN is ranked as the second leading animal disease in China. The annual demand for global rainbow trout is about 5 million tons, with an annual output of approximately 1 million tons and an annual output value of about 100 billion globally. Currently, IHN significantly reduces the breeding efficiency of salmon trout due to the high incidence of rainbow trout IHN disease and the disparity between supply and demand. IHN is distributed in many countries and regions in the world and is mainly spread through the transport of sick fish or contaminated fish eggs between different regions, resulting in outbreaks or local epidemics. The infection was first reported in 1953 in sockeye salmon (*Oncorhynchusnerka*) fry farmed at hatcheries in Washington State and Oregon state, which then rapidly spread along the Pacific Coast to Northern California and Idaho. IHNV was transferred from Alaska to Japan in 1971 through contaminated sockeye salmon eggs and was first isolated from sockeye salmon fingerlings in a hatchery in Hokkaido [10]. In 1987, IHNV was isolated from the yolk sacs of rainbow trout fry in Italy and French rainbow trout fry, and then subsequent IHN outbreaks were reported in Germany, Switzerland, Russia, and other European countries. IHNV mainly infects salmon larvae and fingerlings and can cause severe systemic disease. IHNV can be detected in the hemopoietic tissue of rainbow trout 3 to 4 days after infection. The infected fish exhibit decreased appetite, abnormal swimming actions, sinking to the bottom, floating on water, or wandering in the tank at the early disease stages. The clinical manifestation of the disease includes a change in the color of the fish from light gray to dark gray, black, or dark purple, and ecchymosis is observed on the body surface and the snout. The eyeballs protrude and swell, sometimes exhibiting red color, the gill filaments are pale, and the base of the fin is congested. Abdominal enlargement is observed, and a white or tan tube of stool may appear in the anus [11]. IHNV initially proliferates in hematopoietic tissues, such as the liver, spleen, and kidney, and then infects other internal organs or tissues. Dissection of the infected fish shows significant anemic status, and the hematopoietic tissues, such as the liver, spleen, and kidney, have a light color. The commonly affected tissues are liver tissues, and a large amount of yellowish and muddy, watery, thin mucus is observed in the stomach and intestines.

RETRACTED

Oxidative stress refers to the internal and harmful environment stimulated by reactive oxygen free radicals (ROS) and reactive nitrogen radicals (RNS), resulting in physiological and pathological effects on cells and tissues. Under normal circumstances, the oxidation system and antioxidant system of the body are in dynamic balance [12]. The dynamic balance of the redox reaction is disrupted when oxygen radical productivity exceeds the antioxidant system clearance ability, leading to the accumulation of high levels of reactive oxygen free radicals and, ultimately, oxidative stress. Researchers reported that IHNV mainly infects cells through the clathrin-mediated endocytosis pathway and subsequently triggers activation of the host cellular signaling cascade pathways, including NF-κB signaling pathway [13], autophagy [14], ESCRT pathway [15], and interferon pathway and toll-like receptor signaling pathway [16], which then induces cell damage and promotes viral replication. Studies have been conducted to explore the cellular mechanisms underlying IHNV infection. IHNV alters several cell signaling pathways involved in important physiological functions of the host cells and modulates the intracellular environment to promote its replication process. The aim of the present study was to explore the role of andrographolide as a potential and novel anti-IHNV drug. In addition, the study sought to explore the molecular mechanisms of andrographolide and the targets involved in its function. The findings will provide a theoretical basis for developing novel oral drugs against IHNV.

## 2. Results

### 2.1. Infectious Hematopoietic Necrosis Virus Titer and Growth Curve

The titers of IHNV in EPC cells at 12 h, 24 h, 36 h, 48 h, 60 h, 72 h, 84 h, 96 h, 108 h, 120 h time points were 10^3.36±0.06^, 10^4.30±0.06^, 10^4.63±0.03^, 10^5.42±0.16^, 10^5.87±0.06^, 10^7.32±0.08^, 10^7.67±0.08^, 10^8.27±0.04^, 10^8.29±0.06^, and 10^8.32±0.03^ TCID_50_/0.1 mL, respectively (Figure 1a). The virus titer in the IHNV group was 10^7^ TCID_50_/0.1 mL after 120 h post-infection, which was consistent with the growth curve of IHNV incubated with EPC cells (Figure 1b). The replication efficiency of IHNV on EPC cells was significantly decreased after adding andrographolide compared with the IHNV group (Figure 1b, *p* < 0.05). The 20 μM and 50 μM titers exhibited similar values at 7 d.p.i, 10^4.13±0.04^, and 10^4.36±0.07^ TCID_50_/0.1 mL, respectively. The titer of the virus was significantly lower than the IHNV group (*p* < 0.05) at the same time points, which was consistent with the growth curve of IHNV incubated with EPC after andrographolide treatment.

### 2.2. Cytotoxicity and Rescue Effects of Andrographolide on Infectious Hematopoietic Necrosis Virus-Infected Cells

CPE induced by IHNV on EPC cells was significantly alleviated by andrographolide in a concentration-dependent manner, but cell viability decreased to 66.17 ± 1.46% on day 7 when the concentration was increased to 50 μM (Figure 2a). The cell viability of the 100 μM culture was 31.98 ± 0.72% on day 7 compared with the control group, and significant cell toxicity was observed when the concentration was increased to 100 μM. In this study, 20 μM andrographolide showed the highest rescue effects during IHNV infection.

Different concentrations of andrographolide were used to treat IHNV-infected EPC cells according to the results obtained from the cytotoxicity assay and the morphological observation of IHNV-infected cells. The CPE phenomenon was evident in the IHNV group, with several cells observed shedding in the visual field (Figure 2b). The CPE phenomenon was alleviated by the addition of 5 μM andrographolide, and the number of adherent viable cells increased, but several round-shedding cells were still observed. Cell morphology and indexes were restored to normal status when 20 μM andrographolide was used.

RETRACTED

### 2.3. Andrographolide Upregulates the Expression and Increases the Activity of Antioxidant Enzymes

The expression levels and activities of anti-oxidative enzymes MDA and SOD and the T-AOC in EPC cells after IHNV infection were significantly different from the control group (Figure 3a). MDA level was 196.18 ± 10.97% higher compared with the control group (*p* < 0.01). The level of SOD and T-AOC in the IHNV group decreased to 63.58 ± 1.78% and 66.84 ± 6.12%, respectively, compared with the NC group (*p* < 0.01). Treatment of the cells with 10 μM andrographolide showed significantly lower MDA content compared with the IHNV group, but the level was still higher than the NC group (*p* < 0.01). T-AOC level and the activity of SOD activity were significantly higher after treatment with andrographolide, but the levels were still lower than the NC group (*p* < 0.01). SOD activity and T-AOC level were significantly restored after treatment with 20 μM andrographolide compared with the IHNV group, and the levels were higher than the control group (*p* < 0.05), whereas MDA content was restored to the normal level (*p* > 0.05). These findings indicated that IHNV infection inhibits anti-oxidative enzymes and anti-oxidative reactions. Andrographolide alleviates the oxidative damage induced by IHNV infection.

### 2.4. Andrographolide Decreases the Levels of Reactive Oxygen Species Induced by Infectious Hematopoietic Necrosis Virus Infection

DCFH is not fluorescent and does not permeate the cell membrane, so the probe rapidly accumulates in the cell. However, intracellular reactive oxygen species oxidize non-fluorescent DCFH to produce fluorescent DCF. The intensity of green fluorescence is proportional to the amount of reactive oxygen species. Reactive oxygen species cause damage mainly by oxidation of proteins and unsaturated fatty acids, ultimately damaging organs and tissues. The present study showed IHNV infection-induced accumulation of high levels of intracellular ROS compared with the control group (Figure 3b, *p* < 0.01). The ROS level in the IHNV group decreased after treatment with 10 μM andrographolide, and the ROS level was restored to normal level when 20 μM andrographolide was used (*p* < 0.01). The fluorescence intensity of cells after IHNV infection increased from 0.98 ± 0.02 to 7.63 ± 0.09 (Figure 3c, *p* < 0.01). The fluorescence intensity of the positive ROS staining decreased significantly after andrographolide treatment, and the fluorescence intensities of cells after treatment with 10μM and 20μM andrographolide were 1.21 ± 0.02 and 1.00 ± 0.03, respectively. These results indicate that andrographolide inhibited the accumulation of ROS in cells.

RETRACTED

### 2.5. Andrographolide Inhibits Apoptosis Induced by Infectious Hematopoietic Necrosis Virus Infection

The staining results showed that Hoechst 33342 stained apoptotic cells with a dark blue color, whereas necrotic cells exhibited a red color after staining with PI (Figure 4a). A higher number of apoptotic cells, exhibiting an intense blue color after staining with Hoechst stain, were observed in the IHNV infection group compared with the NC group, whereas few cells showed intense red, a characteristic of necrotic cells after PI staining. The proportion of apoptotic cells decreased after treatment with andrographolide, but there was no significant difference in the number of cells exhibiting an intense red color after treatment with andrographolide. These findings indicate that andrographolide reduced apoptosis induced by IHNV infection, and the mechanism may be related to the modulation of the oxidative stress state. As shown in Figure 4b, the fluorescence intensities of Hoecst 33342 in the NC, IHNV, and IHNV+20 μM groups were 1.01 ± 0.02, 6.30 ± 0.05, and 1.10 ± 0.11, respectively, indicating that IHNV infection induced apoptosis of cells (Figure 4b, *p* < 0.05). Analysis of the cells showed that some nuclei were fragmented and had a crescent shape. The PI fluorescence intensities of the NC, IHNV, and IHNV+20 μM groups were 0.97 ± 0.01, 1.66 ± 0.12, and 0.91 ± 0.05, respectively. These results show that andrographolide alleviates apoptosis and necrosis induced by IHNV infection.

### 2.6. Prediction of Interactions between Infectious Hematopoietic Necrosis Virus, Andrographolide, and Host Proteins

The binding energies for interaction between andrographolide and viral proteins G, L, M, N, NV, and P were analyzed by molecular bioinformatics methods (Figure 5). A positive (Etotal > 0) total energy indicates that the interaction requires the external energy supply, whereas a negative total energy (Etotal < 0) indicates that the ligand can easily bind to the protein. The results show that andrographolide binds different viral proteins, among which it has the lowest binding to NV protein. The required binding energy is −282.16 KJ, which can undergo an active reaction, indicating the possibility of andrographolide binding to the viral NV protein. Compared with other proteins, andrographolide binds to the viral M protein at −191.57 KJ, which requires the highest energy, indicating that andrographolide is the least likely to bind to the M protein. The interactions between andrographolide and oxidative stress-related proteins, including *TRXR2*, *TRXR3a*, *TRXR3b*, *NOX1*, *NOX4*, *NOX5*, *SOD1*, *SOD2*, *iNOS*, *GPX1*, *GPX3*, *GPX4a*, *GPX4b*, *GPX7*, *HO-1*, *NRF2*, *Keap1a*, *Keap1b*, *CTSB*, *CTSC*, *CTSD*, *CTSH*, and *CTSK*, were also predicted (Figure 6). Each 3D structure in Figure 6 shows a complex of the receptor protein (NV) and the ligand–protein (target protein). In the figure, each ball represents an atom, the intensity of color represents the distance between the atoms, and the atoms near the active center are presented In pink, whereas the distant atoms are in purple. The figure shows the receptor and ligand–protein binding pose after docking, indicating the receptor-ligand binding energy which is expressed as Etotal. A smaller Etotal value indicates a high possibility of interaction between the NV protein and target proteins. The results show that IHNV infects host CTSs, possibly by binding to NV proteins and inhibiting host cell survival and physiological functions.

RETRACTED

### 2.7. Andrographolide Alleviates Oxidative Stress and Apoptosis Induced by Infectious Hematopoietic Necrosis Virus Infection by Upregulating the Expression of Anti-Oxidative Genes

The expression of anti-oxidative genes, including *NRF2*, *HO-1*, *GPX3*, *CAT*, *TRXR2*, *TRXR3a*, and *TRXR3b*, was significantly downregulated in the IHNV group compared with the NC group (Figure 7, *p* < 0.01). The expressions of these genes were significantly upregulated after treatment with andrographolide compared with the IHNV group that was not treated with andrographolide (*p* < 0.01). The PI staining results in the previous section showed that IHNV infection induced necrosis, so we evaluated the expression levels of genes implicated in the necrotic pathway. The expression levels of *RIPK1, RIPK3,* and *MLKL* were significantly upregulated after IHNV treatment compared with the NC group (*p* < 0.05). The results of the gene expression analyses were consistent with the trend of PI staining presented in Figure 4. The expression of *CTSB*, *CTSC*, *CTSK*, *CTSZ*, *BAX*, *Cytc*, *Caspase3*, *Caspase8*, and *Caspase9* genes implicated in the apoptosis pathway was significantly upregulated after IHNV infection compared with the control group (*p* < 0.05). On the contrary, the expression of *BCL2* was significantly downregulated after IHNV infection (*p* < 0.01). The expression of anti-oxidative stress genes was upregulated after andrographolide treatment compared with the IHNV group not treated with andrographolide (*p* < 0.01), whereas the expression of apoptotic genes except *BCL2* was downregulated (*p* < 0.05). The expression of necrosis-related genes was significantly inhibited after treatment with andrographolide (*p* < 0.05). The expression levels of *GAPDH* and tubulin beta genes were detected and used as reference genes (Figures S2 and S3).

RETRACTED

## 3. Discussion

IHNV is the pathogen that causes acute fish IHN. This infection is associated with a mortality rate ranging from 90 to 100% in rainbow trout. The World Organization for Animal Health (OIE) listed IHN as an animal disease that must be evaluated during the import and export of fish products due to the significant economic losses caused by IHN to the salmon trout farming industry globally. Currently, vaccines are primarily used for the prevention and control of IHN [17]. Conventional IHN vaccines mainly include inactivated vaccines, live attenuated vaccines, and recombinant vaccines. Recombinant IHN vaccines include subunit vaccines, synthetic peptide vaccines, and nucleic acid vaccines [18]. The vaccine development process takes a long time, the administration procedure is complicated, and the application in the actual breeding environment has drawbacks, thus limiting the use of vaccines for the control of IHN. Therefore, there is an urgent need to identify and design immune-enhancing and antiviral drugs or compounds with simple handling that can be administered through the oral route.

Andrographolide is a diterpenoid lactone with various biological effects, including anti-inflammatory [19], antibacterial [20], and anti-cancer activities, and it exhibits protective effects against the liver, heart, and nervous system. In addition, andrographolide improves the production in livestock and poultry, promotes intestinal health, enhances immunity, is natural, pollution-free, and has no toxic side effects, so it is currently used as a feed additive. Clinical studies indicate that andrographolide can be used to treat various conditions, such as osteoarthritis, upper respiratory diseases, and multiple sclerosis. Previous findings indicate that administration of andrographolide can modulate glucose metabolism and inhibit inflammatory responses and apoptosis [21]. Recent in vitro studies showed that paniculata lactone could be used to treat the new coronavirus [22] and could also inhibit the secretion of Hepatitis B Virus surface antigen [23]. Andrographolide is a widely available compound in the natural environment, so it is easily accessible and not costly. The findings In this study showed that 10 μM concentration exhibited antiviral effect and antiviral effects, with 20 μM andrograpanolide showing the highest effect. In the present study, we observed that andrographolide inhibited the growth of IHNV in cells and alleviated the damage caused by IHNV infection. However, the molecular mechanism of andrographolide against viruses, especially the IHNV, is still unclear, so we conducted this study to explore the mechanism underlying the activity of this compound against IHNV.

RETRACTED

The factors that induce oxidative stress are mainly divided into two categories: endogenous factors (such as aerobic respiration, enzymatic reaction, and phagocytosis) and exogenous factors (including environmental overcooling, overheating, toxin pollution, drug treatment, and disease state). Body homeostasis is disrupted by internal and external factors that affect lipids, proteins, and nucleic acids and eventually cause oxidation of biological molecules, abnormal organ structure, and physiological dysfunction. In addition, the occurrence of oxidative stress is associated with viral infection. Different viruses use different mechanisms to induce oxidative stress. For instance, studies reported that the Sendai virus induced oxidative stress for the first time in 1979 [24]. Several studies report oxidative stress in various organs, including immune organs, after an attack by viral infections [25]. Infection of tissues with influenza, rhinovirus, and several other viruses promotes the production of excessive ROS [26,27]. Most hosts with viral infection present with chronic oxidative stress, which affects the pathogenesis of the disease through impaired immunity, apoptosis, inflammatory response, and organ and tissue dysfunction [28]. Therefore, hosts must maintain a stable redox balance to mount a rapid immune response upon viral entry. Production of excessive ROS leads to the development of oxidative stress, which causes cellular and tissue damage. Previous research on IHNV mainly focused on viral virulence, mechanisms of immune decline, and vaccine development. In the present study, we observed that the antioxidant capacity of EPC cells decreased after IHNV infection. The results showed that the activities of anti-oxidative enzymes, SOD, and T-AOC significantly decreased, whereas the content of MDA increased after IHNV infection. However, cell viability and content of antioxidant enzymes were significantly restored after treatment with andrographolide. Furthermore, the proportion of positively stained cells significantly increased after IHNV infection, indicating higher intracellular ROS. The level of ROS-positive cells decreased after andrographolide treatment, which was consistent with the contents of an antioxidant enzyme. These results indicate that IHNV infection reduces the activity of cellular antioxidant enzymes and induces the accumulation of ROS, leading to cell damage.

RETRACTED

Production of ROS induces the occurrence of oxidative stress, which, in turn, causes ultrastructural changes, cell damage, and adverse changes through activation of apoptosis, necrosis, pyroptosis, and ferroptosis cell death pathways. High expression levels of genes associated with oxidative stress induce apoptosis, necrosis, or ferroptosis. The expression levels of *NRF2*, *HO-1*, *GPX3*, *CAT*, *TRXR2*, *TRXR3*, and *TRXR3b*, which are proteins associated with oxidative stress, were determined in the present study, and the results showed differential expression of these proteins between the infected group and the control group. In the present research, apoptosis features were observed in the IHNV infection group, and a high number of differentially expressed genes implicated in apoptosis were observed between the infected and control groups. In this study, we examined the expression levels of key genes involved in cell death-related signaling pathways and observed that the apoptosis pathway was significantly activated by IHNV infection. The proportion of apoptotic and necrotic positive cells with high fluorescence intensity increased significantly after IHNV infection (*p* < 0.01), which was consistent with the results on accumulation of ROS and oxidative stress-related gene expression levels after IHNV infection. However, the addition of andrographolide alleviated the damaging effects of IHNV on cells, downregulated the expression of genes that promote oxidative stress, inhibited the production of ROS, and promoted the anti-oxidative activity by upregulating expression of antioxidant genes, thus inhibiting the occurrence of apoptosis.

In summary, IHNV infection induces a decrease in the activity of antioxidant enzymes and accumulation of ROS, leading to increases in *CTSK* expression, which further inhibits the expression of *BCL2*, promotes the formation of CytC-induced apoptosome, and ultimately induces the occurrence of apoptosis. Andrographolide treatment effectively alleviates the apoptosis caused by the increased expression of genes that promote the occurrence of oxidative stress and ROS accumulation. The present findings provide a theoretical and practical basis for improving the antioxidant capacity and disease resistance of fish during breeding and lay a foundation for subsequent research on the protective effects of this compound.

## 4. Materials and Methods

### 4.1. Cells, Virus, and Reagents

The epithelioma papulosum cyprini (EPC) cell line (CRL-2872, ATCC), which was stored in liquid nitrogen, was used in this study. The cells were retrieved and immediately placed in a preheated water bath at a constant temperature of 30 °C, with shaking from time to time. This step was performed to melt the cells for 1–2 min to avoid recrystallization and cell damage by the ice crystals. The cells were centrifuged at 1000 g/min for 2 min to coagulate them. The cell freeze solution was carefully sucked out, and 1 mL cell culture solution (MEM basic medium (Thermo Fisher Scientific, Waltham, MA, USA) + 10% fetal bovine serum (Gibco BRL, Grand Island, NY, USA) +100 units/mL of penicillin and streptomycin (Gibco, Grand Island, NY, USA) was added to the cells. Subsequently, the cells were transferred into a sterile T-25 cell culture bottle, and 4 mL of cell culture solution was added. The EPC cells were incubated in a carbon dioxide incubator at 25 °C, 5% CO_2_ (Carbon dioxide was purchased from Harbin Qinghua gas(Harbin, China), whose purity is over 99.9%). After 2–3 days, the original culture medium was discarded after the cells were evenly coated with a single layer of cells, and the cells were digested with 1 mL 0.25% trypsin for about 1 min. Fresh cell culture medium was added, and the cells were gently blown and mixed and then transferred to a new T-25 cell culture bottle for 1:2 continuous passage culture. IHNV-Sn1203 (GenBank No.: KC660147.1) was isolated from a diseased rainbow trout and stored in our laboratory. The characterization of IHNV was conducted as described in a previous study [9]. Andropanolide, which was purchased from Meilunbio (MB2185-1, Dalian, China), was dissolved with 1 mL DMSO and filtered to obtain 500 μM stock solution, packaged and frozen at −20 °C. The solution was diluted before use according to the experimental requirements.

RETRACTED

### 4.2. Infectious Hematopoietic Necrosis Virus Infection and Sample Collection

EPC cells were seeded at a density of 2 × 10^4^ cells per well in 96-well plates, whereas cells were cultured at a density of 5 × 10^4^ cells per well. EPC cells were infected with 0.1 multiplicity of infection (MOI) of IHNV for 1 h, then washed with PBS and cultured in MEM containing 2% FBS at 15 °C and 5% CO_2_ to establish the IHNV infected model. Cells in the IHNV infected group (IH group) and IHNV uninfected group (NC group) were obtained after 72 h post-infection (pi). Total RNA was extracted from the cells using a PrimeScript RT reagent kit with a DNA Eraser (TaKaRa, Shiga, Japan) kit according to the manufacturer’s instructions. The quality of RNA was determined using a NanoDrop 1000 Spectrophotometer (Thermo Fisher Scientific, Waltham, MA, USA). The Epicenter Ribo-Zero Gold kit (Illumina, San Diego, CA, USA) was used to eliminate ribosomal RNA (rRNA) from total RNA, and reverse transcription of the RNA was conducted to obtain cDNA templates.

RETRACTED

### 4.3. Cytotoxicity Assays

24 h after cells were seeded in a 96-well plate, cells were treated with gradient con-centration of andrographolide for 7 days post-infection. After the dilution of andrographolide to the final concentration by laying the cells in 96-well plates for 24 h, the culture medium was discarded, and PBS was used to wash the plate twice. A final concentration of 5 μM was subsequently added to each well. 5 μM, 10 μM, 20 μM, 50 μM, 100 μM cell culture medium containing andrographolide were subsequently cultured for 7 consecutive days. At every 24 h intervals, the culture medium was discarded before adding 10 μL CCK8 solution to each group of cells (to avoid creating bubbles and affecting OD reading). The plates were placed back into the incubator and incubated for 2 h. The absorbance was measured at 450 nm by using a microplate reader.

### 4.4. Determination of Virus Titer and Mapping of Virus Growth Curve

The intracellular virus titers were determined using the Reed–Muench method and the plaque method. All the experiments in this section were conducted in triplicates for each group. For the virus titer determination, 0.1 mL of virus suspension was obtained and continuously diluted 10 times with MEM maintenance medium. The virus suspensions with different concentrations were inoculated into EPC cells in 96-well plates. Each sample was connected to 8 holes and cultured at 15 °C for 7 days. The holes exhibiting the CPE phenomenon were counted, and the TCID_50_ of IHNV was calculated according to our previous study [9].

The virus suspension was diluted to 100 TCID_50_/0.1 mL using MEM maintenance medium, and EPC cells were inoculated with 1 mL of the virus suspension using a cell culture dish with a diameter of 35 mm. The virus suspension was collected in a petri dish every 24 h, and the virus was harvested twice by freezing and thawing. The titer of each strain was measured at different time points using the Reed–Muench method, and a growth curve was drawn.

### 4.5. Determination of Antioxidant Enzyme Activities and Contents

The NC, IHNV, IHNV+10 μM andrographolide and IHNV+20 μM andrographolide groups samples were ground with an electric homogenizer for subsequent enzyme analysis. The total antioxidant capacity (T-AOC) and activities of free radical scavenging enzymes, such as superoxide dismutase (SOD) and malondialdehyde (MDA) (indexes of oxidative damage), were determined using the respective commercial anti-oxidative assay kits (Jiancheng Biotechnology Research Institute, Nanjing, China) to compare anti-oxidative abilities of NC, IHNV, IHNV+10μM andrographolide and IHNV+20 μM andrographolide groups. The assays were performed in our laboratory using SpectraMax^®^ i3x multi-mode microplate readers (Molecular Devices, Shanghai, China) following the manufacturer’s instructions.

RETRACTED

### 4.6. Determination of Reactive Oxygen Species in EPC Cell Lines

The ROS kit (S0033S) (Beyotime Biotechnology, Nanjing, China) was used to determine the ROS levels in EPC cell lines. DCFH-DA (ROS fluorescent probe) was diluted to a final concentration of 10 μmol/L at a ratio of 1:1000 using a basic MEM medium to stain the cells in a 96-well plate. The cells were seeded into a cell culture plate and cultured. The cell culture medium was discarded using a pipette, and the cells were washed with PBS buffer preheated at room temperature. Subsequently, DCFH-DA was incubated in a cell incubator at 37 °C for 20 min to achieve 1 mL/well. The cells were washed, and samples were loaded with probes in situ that could be observed directly with a laser confocal microscope, or cells could be collected and examined with a fluorescence spectrophotometer, a fluorometer, or a flow cytometry. Samples loaded with probes after cell collection can be examined with a fluorescence spectrophotometer, fluorescent enzyme spectrometer, or flow cytometry or directly observed with a confocal laser microscope. Photographed away from light, the ROS levels were recorded. A fluorescence microscope with an excitation wavelength of 488 nm and an emission wavelength of 525 nm was used for the determination of ROS levels.

### 4.7. Reverse Transcription Quantitative Polymerase Chain Reaction

Total RNA was extracted from EPC cells incubated with different IHNV strains using TRIzol reagent (Thermo Fisher Scientific, Waltham, MA, USA) according to the manufacturer’s instructions following a method described in previous research [29]. The RNA was reverse transcribed into cDNA using the HiScript III 1st Strand cDNA Synthesis Kit (+gDNA wiper) (R312-01, Vazyme, Nanjing, China). Expression levels of IHNV component proteins L and G were determined to validate infection of IHNV. Expression levels of oxidative stress-related genes, including TRXR2, TRXR3a, TRXR3b, GPX3, CAT, HO-1, iNOS, Keap1a, and Keap1b, in EPC cells were also detected. In addition, the expression levels of apoptosis-related genes, including BAX, BCL2, Cytc, Caspase3, Caspase6, Caspase7, Caspase8, Caspase9, CTSB, CTSC, CTSD; necrosis pathway genes RIPK1, RIPK3, MLKL, were determined. The housekeeping genes β-actin, GAPDH, and tubulin beta were used as reference genes in the present study. Detailed information on primers used for the qRT-PCR assays is presented in Supplementary Table S1. 10 μL reaction mixtures were incubated in the Applied Biosystems™ QuantStudio™ 6 Hex System (Thermo Fisher Scientific, USA). The reaction mix was mixed as recommended in the instructions for the HiScript III RT SuperMix qPCR (R323-01, Vazyme, Nanjing, China) kit. The PCR procedure was designed as follows: 1 cycle at 95 °C for 30 s and 35 cycles at 95 °C for 15 s and 60 °C for 30 s. The relative abundance of the mRNAs was analyzed using the Pfaffl method [30,31]. The relative expressions of the gene transcripts were determined using the comparative cycle threshold (Ct) method (2^−ΔΔCt^).

RETRACTED

### 4.8. Prediction of Interactions between Andrographolide, Infectious Hematopoietic Necrosis Virus Proteins, and Anti-Oxidative Proteins

Molecular docking studies were conducted to explore the interaction between andrographolide and IHNV proteins. The three-dimensional structure of the target protein was retrieved from the RCSB PDB database https://www.rcsb.org/. For proteins that had no PDB file, the protein sequence was retrieved from NCBI using the species and protein name. Subsequently, the sequence was used to generate 3D protein structure models using Modeller 10.4 software through comparative modeling. Interactions between NV protein and anti-oxidative relative proteins were achieved using Modeller, RCSB PDB database, and Hex8.0.0.

Hex 8.0.0 is a software to predict interactions between proteins/small molecules and proteins, which is used for molecular docking in this study. Hydrogen atoms and charges were added to andrographolide, the target protein structures, and then molecular docking was performed. The docking poses and the interactions between IHNV and andrographolide were analyzed using the Discovery Studio tool.

### 4.9. Determination of Cell Apoptosis Using Hoechst 33342/PI Apoptosis Kit

Hoechst 33342 and Propidium Iodide (PI) double-stained kits (Biosharp, Hefei, China) were used to detect positively stained dead cells in NC, IHNV, and IHNV+Andro groups. The cells were double-stained with Hoechst 33342 and Propidium Iodide (PI). The nuclear fluorescent dye Hoechst 33342 can penetrate the cell membrane and release blue fluorescence after embedding on double-stranded DNA. The membrane of cells in the control group exhibited a light blue color. Hoechst 33342 penetrated apoptotic cells significantly more than normal cells due to the higher permeability of the cell membrane of apoptotic cells. As a result, the fluorescence intensity of apoptotic cells was higher than that of normal cells. Living cells were resistant to the PI dye, whereas the integrity of the cell membrane of necrotic cells was lost at an early stage and was easily stained by PI dye. Fluorescence microscopy was performed after double staining, and the normal cells exhibited light blue/light red (Hoechst 33342+/PI+) color, whereas apoptotic cells exhibited intense blue/light red (Hoechst 33342++/PI+) color. Necrotic cells showed light blue/intense red (Hoechst 33342+/PI++) color.

RETRACTED

### 4.10. Statistical Analysis

Data were expressed as mean ± standard deviation (SD) and analyzed using SPSS 19.0 (SPSS Inc., Chicago, IL, USA) software. The significance level was set at 0.05. A two-tailed unpaired *t*-test was used in all tests except for the generation of survival curves. The survival curves were constructed using a log-rank test and a 95% confidence interval. GraphPad Prism 8 was used to generate figures and graphs. 

## Figures and Tables

**Figure 1:** Titers and growth curves of IHNV incubated with EPC cells at different time points. (**a**) Viral titers in EPC cells at different time points; (**b**) Growth curves of IHNV growing in EPC cells at different time points.

**Figure 2:** Effect of different concentrations of andrographolide on IHNV infected/uninfected cells. (**a**) Effect of different concentrations of andrographolide on cell viability. (**b**) Antiviral effects of different concentrations of andrographolide on IHNV. The scale is 200 μm.

**Figure 3:** Effect of andrographolide and IHNV infection on the antioxidant capacity of EPC cells. (**a**) Effect of andrographolide and IHNV infection on cell viability and the expression levels of antioxidant enzymes. * Represents significant differences compared with the NC group (*p* < 0.05). # Represents significant differences between IHNV and IHNV+20 Μm groups (*p* < 0.05); (**b**) The effects of IHNV infection and andrographolide treatment on intracellular ROS levels as determined by fluorescent staining. The white arrows represent cells with positive staining. The scale is 200 μm; (**c**) The statistical analysis results of ROS fluorescence staining, * representing a significant difference compared with the NC group (*p* < 0.05); # represents significant differences between groups (*p* < 0.05).

**Figure 4:** Effect of andrographolide and IHNV infection on cell death. (**a**) Apoptotic cells are colored in bright blue, and necrotic cells are colored in red. The white arrows represent cells with positive staining. The scale is 200 μm. (**b**) The statistical analysis results of Hoechst33342/PI fluorescence staining, * representing a significant difference compared with the NC group (*p* < 0.05).

**Figure 5:** Prediction of the binding between andrographolide and IHNV viral proteins. The interactions were assessed by the numerical analysis of binding energy (Etotal), whereby Etotal < 0 indicated binding between the ligand and protein target. A smaller Etotal value indicates a higher possibility of binding. The structures formed by the red-green globules represent andrographolide, and the 3D structure composed of the remaining color pellets is the viral protein of IHNV.

RETRACTED

**Figure 6:** Prediction of interactions between host proteins and NV proteins of IHNV. The binding efficiency was determined by the numerical analysis of the Etotal value, with Etotal < 0 indicating high binding affinity. A smaller value of Etotal indicates a higher binding affinity between the ligand and target.

**Figure 7:** Effect of IHNV and andrographolide on expression levels of oxidative stress, apoptosis, and necrosis pathway genes. (**a**) Effect of andrographolide on genes coded IHNV virus proteins. (**b**) Effect of andrographolide on the expression of genes involved in necroptosis pathway. (**c**) Effect of andrographolide on the expression of genes related to oxidative stress. (**d**) Effect of andrographolide on the expression of genes involved in apoptosis. * Represents differentially expressed genes compared with the NC group (*p* < 0.05).

## Data Availability

The data presented in this study are available in the article and supplementary materials.

## Supplementary Materials

The following supporting information can be downloaded at https://www.mdpi.com/article/10.3390/ijms25010308/s1.

## References

[1] Gao J., Peng S., Shan X., Deng G., Shen L., Sun J., Jiang C., Yang X., Chang Z., Sun X. (2019). Inhibition of AIM2 inflammasome-mediated pyroptosis by Andrographolide contributes to amelioration of radiation-induced lung inflammation and fibrosis. Cell Death Dis..

[2] Ren X., Xu W., Sun J., Dong B., Awala H., Wang L. (2021). Current Trends on Repurposing and Pharmacological Enhancement of Andrographolide. Curr. Med. Chem..

[3] Kumar G., Singh D., Tali J.A., Dheer D., Shankar R. (2020). Andrographolide: Chemical modification and its effect on biological activities. Bioorg. Chem..

[4] Van Chien T., Van Loc T., The Anh N., Van Sung T., Phuong Thao T.T. (2023). Cytotoxic and Anti-Inflammatory Activity of 3,19-Isopropylidene-/Arylidene-Andrographolide Analogs. Chem. Biodivers..

[5] Malat P., Ekalaksananan T., Heawchaiyaphum C., Suebsasana S., Roytrakul S., Yingchutrakul Y., Pientong C. (2021). Andrographolide Inhibits Lytic Reactivation of Epstein-Barr Virus by Modulating Transcription Factors in Gastric Cancer. Microorganisms.

[6] Wang X.R., Jiang Z.B., Xu C., Meng W.Y., Liu P., Zhang Y.Z., Xie C., Xu J.Y., Xie Y.J., Liang T.L. (2022). Andrographolide suppresses non-small-cell lung cancer progression through induction of autophagy and antitumor immune response. Pharmacol. Res..

RETRACTED

[7] Yadav R.P., Sadhukhan S., Saha M.L., Ghosh S., Das M. (2022). Exploring the mechanism of andrographolide in the treatment of gastric cancer through network pharmacology and molecular docking. Sci. Rep..

[8] Xu L.M., Liu M., Zhao J.Z., Cao Y.S., Yin J.S., Liu H.B., Lu T. (2014). Epitope mapping of the infectious hematopoietic necrosis virus glycoprotein by flow cytometry. Biotechnol. Lett..

[9] Zhao J.Z., Xu L.M., Zhang Z.Y., Liu M., Cao Y.S., Yin J.S., Liu H.B., Lu T.Y. (2019). Recovery of recombinant infectious hematopoietic necrosis virus strain Sn1203 using the mammalian cell line BHK-21. J. Virol. Methods.

[10] Nishizawa T., Kinoshita S., Kim W.S., Higashi S., Yoshimizu M. (2006). Nucleotide diversity of Japanese isolates of infectious hematopoietic necrosis virus (IHNV) based on the glycoprotein gene. Dis. Aquat. Organ..

[11] Enzmann P.J., Castric J., Bovo G., Thiery R., Fichtner D., Schütze H., Wahli T. (2010). Evolution of infectious hematopoietic necrosis virus (IHNV), a fish rhabdovirus, in Europe over 20 years: Implications for control. Dis. Aquat. Organ..

[12] Wu D., Dasgupta A., Read A.D., Bentley R.E.T., Motamed M., Chen K.H., Al-Qazazi R., Mewburn J.D., Dunham-Snary K.J., Alizadeh E. (2021). Oxygen sensing, mitochondrial biology and experimental therapeutics for pulmonary hypertension and cancer. Free Radic. Biol. Med..

[13] Hoferer M., Akimkin V., Skrypski J., Schütze H., Sting R. (2019). Improvement of a diagnostic procedure in surveillance of the listed fish diseases IHN and VHS. J. Fish Dis..

[14] Wu Y., Guo M., Hua X., Duan K., Lian G., Sun L., Tang L., Xu Y., Liu M., Li Y. (2017). The role of infectious hematopoietic necrosis virus (IHNV) proteins in the modulation of NF-κB pathway during IHNV infection. Fish Shellfish Immunol..

[15] Kim J., Cho M., Lim J., Choi H., Hong S. (2022). Pathogenic Mechanism of a Highly Virulent Infectious Hematopoietic Necrosis Virus in Head Kidney of Rainbow Trout (*Oncorhynchus mykiss*) Analyzed by RNA-Seq Transcriptome Profiling. Viruses.

[16] Xu L., Zhao J., Liu M., Kurath G., Breyta R.B., Ren G., Yin J., Liu H., Lu T. (2019). Phylogeography and evolution of infectious hematopoietic necrosis virus in China. Mol. Phylogenet. Evol..

[17] Liu Q., Cai J., Gao Y., Yang J., Gong Y., Zhang Z. (2018). miR-2954 Inhibits PI3K Signaling and Induces Autophagy and Apoptosis in Myocardium Selenium Deficiency. Cell. Physiol. Biochem. Int. J. Exp. Cell. Physiol. Biochem. Pharmacol..

[18] Tang L., Kang H., Duan K., Guo M., Lian G., Wu Y., Li Y., Gao S., Jiang Y., Yin J. (2016). Effects of Three Types of Inactivation Agents on the Antibody Response and Immune Protection of Inactivated IHNV Vaccine in Rainbow Trout. Viral Immunol..

RETRACTED

[19] Ballesteros N.A., Alonso M., Saint-Jean S.R., Perez-Prieto S.I. (2015). An oral DNA vaccine against infectious haematopoietic necrosis virus (IHNV) encapsulated in alginate microspheres induces dose-dependent immune responses and significant protection in rainbow trout (*Oncorrhynchus mykiss*). Fish Shellfish Immunol..

[20] Kim S.Y., Lee K.M., Kim K.H. (2023). Differences between DNA vaccine and single-cycle viral vaccine in the ability of cross-protection against viral hemorrhagic septicemia virus (VHSV) and infectious hematopoietic necrosis virus (IHNV). Vaccine.

[21] Sun S.C. (2017). The non-canonical NF-κB pathway in immunity and inflammation. Nat. Rev. Immunol..

[22] Banerjee M., Parai D., Chattopadhyay S., Mukherjee S.K. (2017). Andrographolide: Antibacterial activity against common bacteria of human health concern and possible mechanism of action. Folia Microbiol..

[23] Li Y., Xiang L.L., Miao J.X., Miao M.S., Wang C. (2021). Protective effects of andrographolide against cerebral ischemia-reperfusion injury in mice. Int. J. Mol. Med..

[24] Peters J.H., Bessler W.G., Schimmelpfeng L. (1979). Adherent cells as targets in mitogenic T-lymphocyte stimulation: Replacement of lymphocyte-bound mitogens by nonmitogenic substances. Immunol. Commun..

[25] Zhao H., Lu L., Peng Z., Chen L.L., Meng X., Zhang C., Ip J.D., Chan W.M., Chu A.W., Chan K.H. (2022). SARS-CoV-2 Omicron variant shows less efficient replication and fusion activity when compared with Delta variant in TMPRSS2-expressed cells. Emerg. Microbes Infect..

[26] Geng C.A., Wang L.J., Zhang X.M., Ma Y.B., Huang X.Y., Luo J., Guo R.H., Zhou J., Shen Y., Zuo A.X. (2011). Anti-hepatitis B virus active lactones from the traditional Chinese herb: Swertia mileensis. Chemistry.

[27] Ishii H., Nakamura-Hoshi M., Shu T., Matano T. (2022). Sendai virus particles carrying target virus glycoproteins for antibody induction. Vaccine.

[28] Jones D.P. (2006). Redefining oxidative stress. Antioxid. Redox. Signal..

[29] Chen Y., Li J., Zhou Y., Feng Y., Guan X., Li D., Ren X., Gao S., Huang J., Guan X. (2019). The role of infectious hematopoietic necrosis virus (IHNV) proteins in recruiting the ESCRT pathway through three ways in the host cells of fish during IHNV budding. Fish Shellfish Immunol..

[30] Li S., Xie H., Yan Z., Li B., Wu P., Qian X., Zhang X., Wu J., Liu J., Zhao X. (2019). Development of a live vector vaccine against infectious hematopoietic necrosis virus in rainbow trout. Fish Shellfish Immunol..

[31] Enzmann P.J., Kurath G., Fichtner D., Bergmann S.M. (2005). Infectious hematopoietic necrosis virus: Monophyletic origin of European isolates from North American genogroup M. Dis. Aquat. Organ..

